This article has been retracted.

# Asthmatic Airway Vagal Hypertonia Involves Chloride Dyshomeostasis of Preganglionic Neurons in Rats

**DOI:** 10.3389/fnins.2020.00031

**Published:** 2020-01-31

**Authors:** Ding He, Hong Chen, Ming Zeng, Chunmei Xia, Jin Wang, Linlin Shen, Danian Zhu, Yonghua Chen, Jijiang Wang

**Affiliations:** Department of Physiology and Pathophysiology, School of Basic Medical Sciences, Fudan University, Shanghai, China

**Keywords:** Na^+^-K^+^-2Cl^–^ co-transporter 1/K^+^-Cl^–^ co-transporter 2, asthma, microglia, bumetanide, airway vagal preganglionic neuron, minocycline

## Abstract

Airway vagal hypertonia is closely related to the severity of asthma; however, the mechanisms of its genesis are unclear. This study aims to prove that asthmatic airway vagal hypertonia involves neuronal Cl^–^ dyshomeostasis. The experimental airway allergy model was prepared with ovalbumin in male adult Sprague-Dawley rats. Plethysmography was used to evaluate airway vagal response to intracisternally injected γ-aminobutyric acid (GABA). Immunofluorescent staining and Western-blot assay were used to examine the expression of microglia-specific proteins, Na^+^-K^+^-2Cl^–^ co-transporter 1 (NKCC1), K^+^-Cl^–^ co-transporter 2 (KCC2) and brain-derived nerve growth factor (BDNF) in airway vagal centers. Pulmonary inflammatory changes were examined with hematoxylin and eosin staining of lung sections and ELISA assay of ovalbumin-specific IgE in bronchoalveolar lavage fluid (BALF). The results showed that histochemically, experimental airway allergy activated microglia, upregulated NKCC1, downregulated KCC2, and increased the content of BDNF in airway vagal centers. Functionally, experimental airway allergy augmented the excitatory airway vagal response to intracisternally injected GABA, which was attenuated by intracisternally pre-injected NKCC1 inhibitor bumetanide. All of the changes induced by experimental airway allergy were prevented or mitigated by chronic intracerebroventricular or intraperitoneal injection of minocycline, an inhibitor of microglia activation. These results demonstrate that experimental airway allergy augments the excitatory response of airway vagal centers to GABA, which might be the result of neuronal Cl^–^ dyshomeostasis subsequent to microglia activation, increased BDNF release and altered expression of Cl^–^ transporters. Cl^–^ dyshomeostasis in airway vagal centers might contribute to the genesis of airway vagal hypertonia in asthma.

## Introduction

The airway vagal nerves provide the primary cholinergic control to the airway (Canning, 2006). Airway vagal preganglionic neurons (AVPNs), as the final efferent neurons through which the brain controls airway vagal activity, are primarily located in the dorsal motor nucleus of the vagus, the compact and external formation of the nucleus ambiguus (NA), and the intermediate zone between the dorsal motor nucleus of the vagus and NA (Jordan, 2001; Haxhiu et al., 2005; Canning, 2006). AVPNs in the external formation of the NA (eNA) are thought to be particularly crucial in the vagal control of airway smooth muscle, since only this subset of neurons can cause an increase of airway resistance if experimentally stimulated (Haselton et al., 1992; Kc et al., 2006). AVPNs are intrinsically silent, and their activity relies entirely on their synaptic inputs including excitatory glutamatergic inputs and inhibitory γ-aminobutyric acid (GABA)-ergic and glycinergic inputs (Chen et al., 2007, 2012).

Asthma is characterized by some closely interrelated manifestations including chronic airway inflammation, airway hypersensitivity and airway hyperresponsiveness. While the hypersensitivity of airway vagal afferents constitutes an essential aspect of airway hypersensitivity; the hyperresponsiveness of airway vagal efferent is a critical aspect of airway hyperresponsiveness (Canning, 2006; Szekely and Pataki, 2009; Molfino, 2010; Liccardi et al., 2016). Peripherally, the mechanisms involved in the asthmatic sensitization of airway vagal reflex have been intensively studied. However, it has been well recognized that the onset or exacerbation of asthma is not always accompanied by clear evidence that the already-sensitized airway vagal reflex is activated by certain triggering factors, such as inhalation of irritants and prompt acceleration of airway inflammation. Typical examples are nocturnal and psychological stress-induced onset or exacerbation of asthma. These phenomena raise a possibility that in asthma, the excitability/responsiveness of AVPNs might have also been altered. During night sleep or psychological stress, altered excitability/responsiveness of AVPNs might enable these neurons to trigger the onset or exacerbation of asthma, not only in response to airway stimuli but also, automatically through augmented tonic activity.

Chloride homeostasis determines the direction and amplitude of neuronal response to inhibitory neurotransmitters such as GABA and glycine. In the central nervous system (CNS), neuronal Cl^–^ homeostasis is mainly regulated by Na^+^-K^+^-2Cl^–^ co-transporter 1 (NKCC1) and K^+^-Cl^–^ co-transporter 2 (KCC2). NKCC1 intrude Cl^–^ into, and KCC2 extrude Cl^–^ out of, neurons. Neurons in the NA express both NKCC1 and KCC2. In a developing brain, due to the high-level expression of NKCC1, the response of all types of neurons to inhibitory neurotransmitters and Cl^–^ channel openers is initially excitatory, as it has been shown by a previous study that finds midazolam, an agonist of GABA_A_ type of receptor Cl^–^ channels, caused neuronal excitation in neonatal rats that can be blocked by bumetanide, a selective inhibitor of NKCC1 (Koyama et al., 2013). During the early postnatal development, the expression of NKCC1 is downregulated and that of KCC2 is upregulated in many types of neurons including those in the NA (Liu and Wong-Riley, 2012). In many diseases with neurological disorders such as neuropathic pain (Coull et al., 2005; Pitcher and Cervero, 2010; Dai and Ma, 2014), hyperalgesia (Morgado et al., 2011; Ferrini et al., 2013), epilepsy (Karlocai et al., 2015; Marguet et al., 2015), stress-induced hypertension (Ye et al., 2012; Kim et al., 2013; Choe et al., 2015) and visceral hypersensitivity (Tang et al., 2015), downregulated KCC2 and/or upregulated NKCC1 is found in specific spinal or brain neurons, which contributes to the pathogenesis of these diseases via weakened or converted inhibitory neuronal response to inhibitory neurotransmitters. Moreover, the downregulation of KCC2 and/or upregulation of NKCC1 are closely related to the activation of central microglia and subsequent release of brain-derived neurotrophic factor (BDNF) from activated microglia (Coull et al., 2005; Choe et al., 2015; Tang et al., 2015). These previous studies have further raised the possibility that in chronic inflammatory airway diseases such as asthma, chronic airway inflammation is likely to induce airway vagal disorder via inducing Cl^–^ dyshomeostasis in AVPNs.

This study tests the following hypotheses. In experimental airway allergy, microglia in airway vagal centers are activated, which leads to upregulation of NKCC1 and/or downregulation of KCC2 in putative AVPNs and subsequently, alters the response of airway vagal centers to GABA. Prevention of central microglia activation can attenuate the asthmatic airway vagal hypertonia by the restoration of Cl^–^ dyshomeostasis in putative AVPNs.

## Materials and Methods

### Animals and Ethical Approval

Male Sprague–Dawley rats (seven-week-old, 170–190 g) were purchased from the Experimental Animal Center of the Chinese Academy of Sciences in Shanghai. Before experimental treatments, animals were housed for at least 3 days with food and water supplied *ad libitum*. The feeding room was set at a 12-h light-dark cycle and a temperature of 22 ± 0.5°C. All procedures were following the recommendations of the guidelines for the Care and Use of Laboratory Animals (1996, National Academy of Sciences, Washington, DC, United States), and approved by the Ethical Committee of the Fudan University School of Basic Medical Sciences (Nos. 20110307-060 and 20170223-073). A total of 100 rats were sacrificed. Maximal efforts were made to minimize pain and discomfort to animals.

### Preparation of the Experimental Rat Model of Airway Allergy

The rat model of airway allergy was developed by sensitization injections and inhalation challenge with ovalbumin (OVA). Briefly, 88 rats were assigned into four groups: control group (*n* = 28), OVA sensitization-challenge group (OVA group, *n* = 28), OVA sensitization-challenge plus intraperitoneal minocycline injection group [OVA + MC(ip) group, *n* = 16] and OVA sensitization-challenge plus intracerebroventricular minocycline injection group [OVA + MC(icv) group, *n* = 16]. Animals in OVA, OVA + MC(ip) and OVA + MC(icv) groups were immunized on the 0th day by an intraperitoneal injection of 10 mg OVA (Sigma-Aldrich, grade V) and 2 mg Al(OH)_3_ adjuvant suspended in 1 mL saline. A booster sensitization was given on the 7th day. From the 14th to 28th day, rats survived from the immune injections in each group (28, 28, 16, and 16 rats, respectively) were daily challenged for 30 min in a closed acrylic container (60 cm × 50 cm × 35 cm) with aerosolized 5% OVA (Sigma-Aldrich, grade II) suspension in saline using an ultrasonic nebulizer. Rats in control group underwent identical procedures, except that OVA suspensions for injections or inhalation were taken instead by saline. From the 14th to 28th day, rats in OVA + MC(ip) group were given intraperitoneal injection of minocycline (30 mg/kg) daily before the aerosolization. From the 13th to 28th day, rats in OVA + MC(icv) group were continuously given minocycline solution [172 ng/mL, in artificial cerebral spinal fluid (ACSF)] intracerebroventricularly through an implanted osmotic minipump (see below) at a rate of 0.3 μL/h.

### Implantation of Osmotic Minipump and Infusion Cannula

On the 13th day, rats in OVA + MC(icv) group were heavily anesthetized with continuous inhalation of halothane through a mask and fixed on a stereotaxic apparatus. A midline incision was made on the calvaria. A hole was drilled on the right parietal bone, and the infusion cannula (Kit 2; Alzet Company, Cupertino, CA, United States) was targeted to the right lateral cerebral ventricle (0.8 mm caudal to the bregma; 1.5 mm lateral to the midline; 4 mm below the surface of the skull). An osmotic minipump (Model 2002; Alzet Company) was positioned subcutaneously in the scapular region and attached to the infusion cannula. The cannula was fixed to the skull with bone cement, and the wound was closed and sutured with surgical silk (4.0). Before implantation, the minipump had been filled with minocycline solution and kept at 36°C.

### Intracisternal Injection of Drugs and Plethysmographic Evaluation of Airway Vagal Response

From the 29th to 35th day, 8 rats from control group and 7 rats from OVA group were anesthetized by intraperitoneal injection of the mixture of anesthetics (urethane 0.84 g/kg, α-chloralose 42 mg/kg and borax 42 mg/kg). Intracisternal injection of GABA or bumetanide solution was carried out through the PE-10 catheter inserted into the cisterna magna; and plethysmographic evaluation of airway vagal response was carried out using a pulmonary function analyzing system (AniRes2005, Beijing Biolab Co., Ltd., Beijing, China), as we have described previously (Chen et al., 2019). After the response of pulmonary function to the first-time intracisternal injection of GABA solution (50 μmol/L, 50 μL, in a 20-s period) recovered (usually within 15 min after GABA injection), bumetanide solution (0.5 mmol/L, 40 μL, in a 20-s period) was injected intracisternally, and a second-time injection of GABA solution was carried out 20 min after intracisternal bumetanide injection. To confirm that the pulmonary responses induced by intracisternal injection of GABA were mediated by airway vagal nerves, in another four rats from control group and another five rats from OVA group, subcutaneous injection of atropine sulfate (0.5 mg/kg) was carried out 20 min before the intracisternal injection of GABA (Chen et al., 2019).

### Measurement of OVA-Specific IgE in Blood Serum and Bronchoalveolar Lavage Fluid (BALF)

From the 29th to 35th day, 10 rats from each group were anesthetized by intraperitoneal injection of the mixture of anesthetics mentioned above. After plethysmographic measurement of pulmonary function indices, 200–500 μL peripheral blood was drained from the vena ophthalmica of each rat with glass pipettes, and collected with centrifuge tubes. The thoracic cavity was opened, and the lungs were taken out for collection of BALF. The rat was then perfused transcardially with 150 mL saline and 250 mL 4% paraformaldehyde. The brainstem was taken out and fixed in 4% paraformaldehyde for at least 24 h for further use in immunofluorescent experiments. Blood serum was isolated from the blood by centrifugation at 3000 rpm for 10 min at 4°C and collected. BALF was collected by repeated (five times) washing of the bronchoalveolar space with 6 mL ice-cold isotonic PBS. The BALF was centrifuged at 3,000 rpm for 10 min at 4°C, and the supernatant was collected and stored in −80°C. OVA-specific IgE in BALF and blood serum was measured using a rat ELISA kit (Shanghai Enzyme-linked Biotechnology Co., Ltd., China) in combination with a microplate reader (Infinite M1000 Pro, Tecan, Switzerland) at 450 nm wavelength.

### Western-Blot Assay

From the 29th to 35th day, six rats in each group were anesthetized deeply with inhalation of halothane, and decapitated. The brain was quickly removed and put in a plate placed on ice. The chest was opened, and the middle lobe of the right lungs were isolated and fixed in 4% paraformaldehyde for at least 24 h for further histological examination. The brainstem was quickly dissected and secured on the slicing platform of a freezing microtome (Jung Histocut, Model 820-II, Leica, Germany). Transverse slices were cut rostro-caudally, and the rostral cutting plan was compared with a rat brain atlas (Paxinos et al., 1980). Once the rostral end of the NA was visible, a 4-mm-thick slice was cut. The NA and its surrounding tissue were taken from the slice by punching with a 17-gauge flat-tip needle. The selected tissue sample was homogenized in a RIPA buffer (P0013C, Beyotime Biotechnology, Shanghai, China) containing a protease inhibitor cocktail tablet (Roche Diagnostics GmbH, Mannheim, Germany). The homogenates were then centrifuged at 13,000 rpm for 10 min at 4°C. The supernatant was transferred to a new tube. Protein concentration was detected with a BCA Protein Assay Kit (Beyotime Biotechnology) in combination with a microplate reader (Infinite M200, Tecan, Switzerland). Samples with equal amounts of proteins were separated using 8% or 12% SDS polyacrylamide gel electrophoresis and transferred onto a polyvinylidene difluoride membrane (Millipore, MA, United States). After blocking with 5% non-fat milk for 1 h at room temperature, the filter membranes were incubated overnight at 4°C with primary rabbit antibodies for NKCC1 (D13A9) (1:2000, #8351S, Cell Signaling Technology, United States), KCC2 (1:2000, Abcam, ab49917, United States), Iba1 (1:2000, Abcam, ab178846, United States), BDNF (1:2000, Abcam, ab108319, United States) and mouse antibodies for β-actin (1:2000, AF0003, Beyotime Biotechnology) or GAPDH (glyceraldehyde-3-phosphate dehydrogenase,1:2000, AF0006, Beyotime Biotechnology). After washing, the membranes were incubated with peroxidase-conjugated goat anti-rabbit IgG (1:2000, A0208, Beyotime Biotechnology) or goat anti-mouse IgG (1:2000, A0216, Beyotime Biotechnology) at room temperature for 2 h, and washed three times with TBST. The protein bands were incubated with the BeyoECL Plus (P0018S, Beyotime Biotechnology) and imaged using the ImageQuant LAS 4000 (GE Healthcare, United States). Densitometric data were expressed as the ratio to β-actin or GAPDH protein.

### Histochemical and Morphometric Examination

The fixed lung tissue was embedded in paraffin. Sections of 4–5 μm thickness were cut and stained with hematoxylin and eosin (H&E). The fixed brainstems were placed serially in 20 and 30% sucrose solutions until sinking. Dehydrated brainstems were rapidly frozen in Tissue-Tek (R) OCT compound, secured on the slicing platform of a freezing microtome (Jung Histocut), and sectioned at 30 μm. In immunofluorescent staining, the following primary antibodies were used: goat anti-NKCC1 (1:200, Abcam, ab99558, United States), rabbit anti-KCC2 (1:200, Abcam, ab49917, United States), mouse anti-OX42 (CD11b/c) (1:200, Abcam, ab1211, United States), rabbit anti-BDNF (1:200, Abcam, ab108319, United States). After blocking in 3% donkey serum, the sections were incubated with the primary antibodies overnight at 4°C. Then sections were incubated with the following secondary antibodies for 1 h: donkey anti-rabbit IgG H + L (1:200, Abcam, ab150073, AlexaFluor-488), donkey anti-goat IgG H + L (1:200, Abcam, ab150130, AlexaFluor-555), donkey anti-mouse IgG H + L (1:200, Abcam, ab150105, AlexaFluor-488), donkey anti-rabbit IgG H + L (1:200, Abcam, ab150076, AlexaFluor-594). Slices of the lungs were mounted on glasses, covered with slips, and examined with a light microscope. Brainstem slices were treated with an antifade mounting medium (P0128, Beyotime Biotechnology), covered with slips, and examine with the Leica LSM 510 META confocal microscope.

### Examination of Immunofluorescence

For quantification of KCC2 and NKCC1 immunofluorescence, double fluorescence labeling was captured using frame-channel mode to avoid any cross-talk between the channels. Excitation of the fluorochrome was performed with an argon ion laser set at 488 nm and a helium/neon laser set at 575 nm. In each slice, the optical density of KCC2 and NKCC1 immunofluorescence in a 1-μm-thick optical section was stacked, and signals in a 300 × 300 μm field containing the compact and external portions of the NA were digitized using the Leica 3.3 software. In each rat, three continuous slices across the NA were examined and the optic density ratio of KCC2 and NKCC1 was obtained by average. The intensity and area of OX42 were quantified using the Image-pro plus 6.0 software.

### Data Analysis

Data were expressed as means ±SEM. When data from only two groups were compared, paired or independent *t*-tests was used. When data from more than two groups were compared, one-way ANOVA followed by Tukey correction was used. Shapiro–Wilk test was run before parametric tests to make sure that the data follow a normal distribution. When comparing the data from Western blot essay, the data in control group was set as 1, and the data in other groups were set as the folds of control. Statistic comparisons were performed using the GraphPad Prism 7 software (La Jolla, CA, United States). Significance was set at *p* < 0.05.

## Results

From the 17th to 18th day, all of the rats in OVA group started to show dyspnea, cough, scratching on the nose, drowsiness and decreased movement, which were particularly severe during the 30-min period of daily inhalation challenge, indicating successful inducement of allergic asthma.

### Experimental Airway Allergy Decreased Pulmonary Function and Induced Pulmonary Inflammation, and All of Which Were Attenuated by Intraperitoneal or Intracerebroventricular Minocycline Treatment

Experimental airway allergy caused conspicuous pulmonary inflammation, as shown in rats from OVA group by the infiltration of inflammatory cells around the bronchus and in the interstitium (Figure 1, photos on upper panels), and by the significant increase in the concentration of OVA-specific IgG in BALF (Figure 1A). Experimental airway allergy did not cause significant change of OVA-specific IgG in blood serum (data not shown). In addition, compared with the rats from the control group, rats from the OVA group showed decreased pulmonary function, as was manifested by significant decreases in C_dyn_, PIF, PEF, and significant increases in R_i_ and R_e_ (Figures 1B–F). All of these changes induced by airway allergy were either attenuated or blocked by minocycline in rats of OVA + MC(ip) and OVA + MC(icv) groups (Figure 1) (*n* = 10 in each group). These results demonstrate that in rats of experimental airway allergy, minocycline, whether applied peripherally or intracerebroventricularly, can alleviate the pulmonary inflammation and improve pulmonary function, and suggest that the pulmonary function decrease and pulmonary inflammation might be at least in part due to augmented airway vagal activity, which might be subsequent to activation of central microglia.

**FIGURE 1:** Experimental airway allergy decreased pulmonary function and induced pulmonary inflammation, and all of which were attenuated by intraperitoneal or intracerebroventricular minocycline treatment. The photos on upper panels are H&E staining of lung tissues in control, OVA, OVA + MC(ip) and OVA + MC(icv) groups (examined in ten rats in each group), showing the infiltration of inflammatory cells in rats of OVA group and the alleviation by minocycline in rats of OVA + MC(ip) and OVA + MC(icv) groups. **(A–F)** Bar graphs for the relative concentration of OVA-specific IgE in BALF, inspiratory resistance of the airway (R_i_), expiratory resistance of the airway (R_e_), dynamic compliance of the lungs (C_dyn_), peak inspiratory flow (PIF) and peak expiratory flow (PEF) in rats of control, OVA, OVA + MC(ip) and OVA + MC(icv) groups (*n* = 10 in each group), showing the changes in rats OVA group and the attenuation of the changes by minocycline in rats of OVA + MC(ip) and OVA + MC(icv) groups. *P*-values were obtained from one-way ANOVA followed by Tukey correction.

### Experimental Airway Allergy Caused Activation of Microglia in the Brainstem Particularly in the NA and Nucleus Tractus Solitarius (NTS), Which Was Prevented by Intraperitoneal or Intracerebroventricular Injection of Minocycline

Airway allergy caused activation of microglia in the brainstem, especially in the NA and NTS, as is shown by increased cell count, enlarged cell body and shortened processes in the immunofluorescent staining with anti-OX42 antibody (Figures 2A,B) (examined in five rats in each group), and by increased expression of Iba1 in the NA in Western-blot essay (Figures 2C,D) (examined in six rats in each group). All of the changes of microglia induced by airway allergy was prevented by intraperitoneal or intracerebroventricular treatment with minocycline (Figure 2). These results confirm that experimental airway allergy activated brainstem microglia.

**FIGURE 2:** Experimental airway allergy caused activation of microglia in the brainstem particularly in the NA and nucleus tractus solitarius (NTS), which was prevented by intraperitoneal or intracerebroventricular injection of minocycline. **(A)** Immunofluorescent staining of OX42 in the NTS and NA of rats in control, OVA, OVA + MC(ip) and OVA + MC(icv) groups (examined in five rats in each group). Note that in the NTS and NA of rats in OVA group, the microglia stained by anti-OX42 antibody have increased number and size, and shortened processes, which suggests activation of these cells. **(B)** Summarized data for the optic density of OX42 fluorescence in the NA of rats in different groups, showing the significant increase in rats of OVA group. **(C,D)** Results from Western-blot assay (*n* = 6 in each group) of Iba1, showing the increased expression of Iba1 in the NA of rats in OVA group. All of the changes of microglia were prevented by minocycline treatment in rats of OVA + MC(ip) and OVA + MC(icv) groups. Dashed circles indicate the compact portion of the NA. *P*-values were obtained from one-way ANOVA followed by Tukey correction.

### Experimental Airway Allergy Increased the Expression of NKCC1 and Decreased the Expression of KCC2 in the NA; And Both of Which Were Attenuated by Intraperitoneal or Intracerebroventricular Minocycline

As shown by immunofluorescent staining (Figure 3, upper panels) (examined in five rats in each group), the NA of male adult rats in control group showed positive immunoreactivity of NKCC1 and KCC2, with the most robust NKCC1 immunoreactivity in the soma (particularly the cytosol) of neuron-like cells, and KCC2 immunoreactivity, mainly in the membrane of neuron-like cells and in surrounding fibers. In rats of OVA group, KCC2 immunoreactivity was weakened in the NA, leading to a decreased ratio of the optical density of KCC2 and NKCC1 (Figure 3, bar graph to the right of color photos). Decreased expression of KCC2 in the NA was also obtained by Western-blot assay. Interestingly, Western-blot assay also showed a significant increase in the expression of NKCC1 in the NA (Figure 3, lower panels) (examined in five rats in each group), although this change was not visually obvious in individual neurons in immunofluorescent staining. In rats of OVA + MC(ip) and OVA + MC(icv) groups, the airway allergy-induced changes in the expression of NKCC1 and KCC2 were attenuated by minocycline (Figure 3). These results demonstrate that experimental airway allergy alters the expression of NKCC1/KCC2 in putative AVPNs, which might be able to change the response of AVPNs to inhibitory neurotransmitters by disruption of their Cl^–^ homeostasis. These results also indicate that the alteration in the expression of NKCC1/KCC2 in putative AVPNs is related to activation of central microglia.

**FIGURE 3:** Experimental airway allergy increased the expression of NKCC1 and decreased the expression of KCC2 in the NA; and both of which were attenuated by intraperitoneal or intracerebroventricular minocycline. The photos on upper panels show the immunofluorescent staining of NKCC1 (red) and KCC2 (green) in the NA of rats in control, OVA, OVA + MC(ip) and OVA + MC(icv) groups. Note that NKCC1 immunoreactivity is most active in the soma (particularly the cytosol) of neuron-like cells and KCC2 immunoreactivity is mainly in the membrane of neuron-like cells and in surrounding fibers. The bar graph to the right of the photos shows the optic density ratio of KCC2 and NKCC1 in the NA of rats in different groups (*n* = 5 in each group), which was decreased in rats of OVA group and the decrease was restored in rats of OVA + MC(ip) and OVA + MC(icv) groups. The results of Western-blot assay for NKCC1 and KCC2 are shown on the lower panels, showing the increased expression of NKCC1 and decreased expression of KCC2 in the NA of rats in OVA group, and the changes were prevented by minocycline in rats of OVA + MC(ip) and OVA + MC(icv) groups (*n* = 5 in each group) (note the KCC2 band of this figure and the Iba1 band in Figure 2 were obtained from the same experiment. Therefore, they share the same β-actin band). *P*-values were obtained from one-way ANOVA followed by Tukey correction.

### Experimental Airway Allergy Enhanced the Excitatory Response of Airway Vagal Nerves to Intracisternally Injected GABA, Which Was Attenuated by Intracisternally Pre-injected NKCC1 Inhibitor Bumetanide

To observe whether the altered expression of NKCC1/KCC2 in the NA is able to change the response of putative AVPNs to inhibitory neurotransmitters, the response of airway vagal activity to intracisternally injected GABA solution was then evaluated using plethysmography in eight rats from control group and seven rats from OVA group. In rats of both groups, bolus intracisternal injection of GABA (50 μmol/L, 50 μL, in a 20-s period) increased airway vagal activity, as was manifested by significantly increased inspiratory resistance of the airway (R_i_) and expiratory resistance of the airway (R_e_), and significantly decreased compliance of the lungs (C_dyn_). As illustrated in Figure 4A are the changes in R_i_, R_e_, and C_dyn_ induced by intracisternal injection of GABA in a rat from the OVA group. These pulmonary responses started within 1 min after the injection of GABA, lasted for 3–5 min and were repeatable in individual rats. In comparison, bolus intracisternal injection of 50 μL ACSF did not cause any detectable change. Noticeably, the responses of R_i_, R_e_, and C_dyn_ to GABA injection were much more potent in rats of OVA group, as are shown by the averaged absolute values of R_i_, R_e_ and C_dyn_ in Figures 4B1,B3,B5,C1,C3,C5, and by their changes in percentage of the baselines in Figures 4D1–D3. 20 min after intracisternal pre-injection of bumetanide (0.5 mmol/L, 40 μL, in a 20-s period), an inhibitor of NKCC1 that is commonly used as an diuretic, the responses of R_i_, R_e_, and C_dyn_ induced by GABA injection were converted in rats of control group (Figures 4B2,B4,B6,D1–D3) and attenuated in rats of OVA group (Figures 4C2,C4,C6,D1–D3). Bumetanide alone did not cause any change at the dose used within the period of recording.

**FIGURE 4:** Experimental airway allergy enhanced the excitatory response of airway vagal nerves to intracisternally injected GABA, which was attenuated by intracisternally pre-injected NKCC1 inhibitor bumetanide. **(A)** The changes in inspiratory resistance of the airway (R_i_), expiratory resistance of the airway (R_e_) and compliance of the lungs (C_dyn_) induced by intracisternal injection of GABA in a representative experiment performed in a rat from OVA group, showing the increases in R_i_ and R_e_, and the decrease in C_dyn_. **(B1–B6,C1–C6)** Summarized data for the GABA-induced changes of R_i_, R_e_ and C_dyn_ in 8 rats of control group **(B1–B6)** and 7 rats of OVA group **(C1–C6)** before and after pretreatment with intracisternal bumetanide. **(D1–D3)** The changes in R_i_, R_e_ and C_dyn_ induced by GABA injection are presented as the percentage of the baselines. Note that the GABA-induced changes are significantly more potent in rats of OVA group; and after pretreatment with intracisternal bumetanide, the GABA-induced changes of R_i_, R_e_ and C_dyn_ were converted in rats of control group and attenuated in rats of OVA group. *P*-values in **B1,B3,B5,C1,C3,C5** were obtained from pared *t*-test; *P*-values in **B2,B4,B6,C2,C4,C6** were obtained from one-way ANOVA followed by Tukey correction.

In comparison, in the four rats from control group and the five rats from OVA group that were pretreated with atropine, intracisternal injection of GABA did not cause any change in R_i_, R_e_, and C_dyn_ (Figure 5), suggesting that the GABA-induced changes are mediated by airway vagal nerves. These results demonstrate that experimental airway allergy augments the excitatory response of putative AVPNs to GABA, and further indicate that this augmentation might be due to increased intracellular Cl^–^ of putative AVPNs.

**FIGURE 5:** Pretreatment with atropine abolished the pulmonary responses to intracisternal injection of GABA solution, both in rats of control group and in rats of OVA group. 20 min after subcutaneous injection of atropine sulfate (0.5 mg/kg), intracisternal injection of GABA solution (50 μmol/L, 50 μL, in a 20-s period) did not cause any significant change in C_dyn_, R_i_ and R_e_, either in rats of control group (upper part) or in rats of OVA group (lower part). Raw recordings from representative experiments are shown on the left side; and summarized data are shown as bar graphs on the right side. *P*-values were obtained from paired *t*-test.

For the rats in the control group, putative AVPNs express NKCC1, and intracisternal injection of GABA solution caused increased airway vagal activity, there is a possibility that the expression of NKCC1 and KCC2 in the NA of control rats has also been altered by our experimental procedures. To test this possibility, in four naïve male adult rats of the same age, supplementary immunofluorescent staining experiment was performed. As shown in Supplementary Figure S1, the NA-containing region of naïve adult rats also expresses both NKCC1 and KCC2, but the optic density ratio of KCC2 and NKCC1 is not significantly different with that of rats in control group.

### Experimental Airway Allergy Increased the Content of BDNF in the Brainstem Particularly in the NA, Which Was Prevented by Intraperitoneal or Intracerebroventricular Injection of Minocycline

As shown by immunofluorescent staining with antibodies for both BDNF and OX42 (examined in six rats in each group), in the NA-containing medullary region of rats from both control group and OVA group, positive BDNF immunoreactivity was detected in both cell-like structures and intercellular space, with the most robust immunoreactivity in the compact portion of the NA. Compared with rats from control group, rats from OVA group showed markedly enhanced BDNF immunoreactivity in the NA-containing region (Figure 6, color photos on upper panels). Increased BDNF content in the NA-containing medullary region was also obtained from Western-blot assay (Figure 6, lower panels) (examined in six rats in each group). In rats of OVA + MC(ip) and OVA + MC(icv) groups, the increase of BDNF content was prevented by minocycline (Figure 6). In addition, in rats of OVA group, at least some of the microglia within and around the neuron-aggregating compact portion of the NA were double-stained by antibodies for BDNF and OX42 (Figure 6). However, since AVPNs expressed BDNF as reported (Zaidi et al., 2005), and the double-stained microglia were mostly overlapped with the BDNF-positive AVPNs, it is hard to judge whether these double-stained microglia independently produce BDNF. These results demonstrate that in the NA-containing medullary region of rats from OVA group, the content of BDNF is increased, and suggests that activated microglia might participate in this increase.

**FIGURE 6:** Experimental airway allergy increased the content of BDNF in the brainstem particularly in the NA, which was prevented by intraperitoneal or intracerebroventricular injection of minocycline. The photos on upper panels (20× magnitude) show the immunoreactivity of BDNF and OX42 in the NA-containing region of rats in control, OVA, OVA + MC(ip) and OVA + MC(icv) groups (examined in six rats in each group). Note that in the NA-containing region of rats, positive BDNF immunoreactivity was detected in both cell-like structures and intercellular space, with the strongest immunoreactivity in the compact portion of the NA. And, positive BDNF immunoreactivity was enhanced in rats of OVA group, which was reversed in rats of OVA + MC(ip) and OVA + MC(icv) groups. The lower panels show the expression of BDNF in the NA of rats from different groups obtained from Western-blot assay (*n* = 6 in each group). *P*-values were obtained from one-way ANOVA followed by Tukey correction.

## Discussion

This study found that both NKCC1 and KCC2 are expressed in the NA of rats. The expression of NKCC1 is particularly dense in the soma of neuron-like cells in the compact portion of the NA, which suggests that the concentration of intracellular Cl^–^ in these cells is relatively high. In consistence with this postulation, even in rats of control group, intracisternally injected GABA increased airway vagal activity, which suggests an excitatory response of putative AVPNs. Moreover, in rats from OVA group, the expression of NKCC1 was increased and that of KCC2 was decreased in the NA. Consistently, the excitatory response of airway vagal activity to intracisternally injected GABA was augmented, which was attenuated by intracisternal pretreatment with NKCC1 inhibitor bumetanide. Since AVPNs are densely innervated by GABAergic and glycinergic synaptic inputs (Chen et al., 2007, 2012), this study for the first time demonstrates that experimental airway allergy can change the responsiveness of putative AVPNs to an inhibitory neurotransmitter, which is probably due to the disruption of neuronal Cl^–^ homeostasis. This conclusion is consistent with the findings in previous studies that loop diuretics such as furosemide and bumetanide relieve asthma in both human patients (Inokuchi et al., 2014) and animal models (Polosa et al., 1993; Wang et al., 2011).

It is quite interesting that intracisternally injected GABA increased airway vagal activity in rats from control group. In consistent with this result, the NA-containing region of these rats expresses NKCC1. It thus arises whether the expression of NKCC1 and KCC2 in the NA of rats in control group has also been altered by our experimental procedures. However, this possibility is denied by the results that the NA-containing region of naïve rats also expresses NKCC1; and the optic density ratio of KCC2 and NKCC1 in the NA of naïve rats is not significantly different with that of rats in control group.

Unexpectedly, in this study, intracisternal injection of bumetanide did not cause any significant change of pulmonary function, either in rats of control group or in rats of OVA group. One explanation for these results is that significant relief of asthma by loop diuretics might need the action of these drugs at more sites that are related to pulmonary function, since the expression and asthmatic upregulation of NKCC1 have also been found in alveolar epithelial cells, alveolar type II cells, T lymphocytes in the lungs (Wang et al., 2011) and airway sensory neurons in the nodose ganglion (Mazzone and McGovern, 2008). The other explanation is that Cl^–^ homeostasis, whether in control animals or in asthmatic animals, might only play a minor role in determining the excitability of AVPNs. This second explanation is supported by two facts: one is that the firing of AVPNs has been known to be predominantly triggered by their excitatory inputs (Chen et al., 2007, 2012); the other is that in all types of cells, the resting membrane potential is known to be predominantly determined by K^+^ homeostasis and can only be slightly changed even in cells expressing CI^–^ transporters. Therefore, even in NKCC1-expression cells, the equilibrium potential of Cl^–^ is still close to resting membrane potential, which limits the response of any type of cells to inhibitors of NKCC1 or inhibitory neurotransmitters.

It must be confessed that in the immunohistochemical and Western-blot experiments of this study that detected the expression of NKCC1 and KCC2 in the NA, the nucleus and its surrounding tissue was treated as a whole, thus the results cannot selectively reflect the cytochemical changes of real AVPNs. Similarly, in intracisternal injection experiments, drugs were applied to the whole brainstem but not selectively to AVPNs; therefore, the effects may include polysynaptic actions in the brainstem.

In the brainstem of the rat of OVA group, the changes in the expression of NKCC1 and KCC2 were accompanied by activation of microglia and increased BDNF content, and the increase of BDNF content was particularly prominent in the compact portion of the NA. All of these histochemical changes were prevented by intraperitoneal or intracerebroventricular treatment with minocycline. Since AVPNs themselves are known to synthesize BDNF (Zaidi et al., 2005), and BDNF has been well-recognized to be able to cause upregulation of NKCC1 and/or downregulation of KCC2 (Coull et al., 2005; Choe et al., 2015; Tang et al., 2015), our results suggest that in airway allergy, both BDNF paracrine from activated microglia in the NA and BDNF autocrine from AVPNs might be involved in the alteration of NKCC1/KCC2 expression in putative AVPNs, which subsequently leads to enhanced excitatory response of AVPNs to inhibitory neurotransmitters. However, in the fluorescent staining experiment of this study, since AVPNs expressed BDNF as reported (Zaidi et al., 2005), and the double-stained microglia were mostly overlapped with the BDNF-positive AVPNs, it needs further validation whether activated microglia in the NA participate in the increase of local BDNF content. Allergic peripheral inflammation including airway allergy has been found to cause activation of microglia in the hypothalamus (Win-Shwe et al., 2013), nucleus tractus solitarius (Spaziano et al., 2015) and spinal cord; and activation of spinal microglia plays an important role in the genesis of neuropathic pain (Yamasaki et al., 2016). Our study further supplies evidence that in airway allergy, activated brainstem microglia might be involved in the genesis of asthmatic airway vagal hypertonia via causing neuronal Cl^–^ dyshomeostasis.

Tetracycline derivatives including minocycline have been well known to be able to relieve asthmatic pulmonary inflammation through mechanisms independent of their antibiotic actions (Rempe et al., 2007; Joks et al., 2010; Joks and Durkin, 2011). In this study, intracerebroventricularly applied minocycline, which is far smaller in the dose compared with that applied intraperitoneally, not only reversed the cytochemical alterations in the NA but also attenuated the decrease of pulmonary function and alleviated pulmonary inflammation in rats of airway allergy. These results suggest that in rats of airway allergy, augmented airway vagal activity plays essential roles in the genesis of pulmonary inflammation. These results also indicate that inhibition of central microglia activation alone, via attenuation of airway vagal hypertonia, is sufficient to attenuate asthmatic pulmonary function decrease and alleviate the pulmonary inflammation. However, as antibiotics, tetracycline derivatives have the common side effects of all antibiotics. In particular, gastrointestinal disorders induced by tetracycline derivatives are particularly severe (Gabriel et al., 2018); and the irreversible hyperpigmentation characteristically induced by tetracycline derivatives is particularly unacceptable psychosocially (Voets et al., 2016). Therefore, further study is necessary to identify the endogenous ligands and receptors that cause asthmatic activation of brainstem microglia, so that specific antagonists can be developed.

In summary, this study found that in experimental airway allergy, NKCC1 is upregulated and KCC2 is downregulated in airway vagal centers, leading to augmented excitatory response of putative AVPNs to GABA; and all of the changes induced by airway allergy, including brainstem neurochemical, airway vagal functional, pulmonary functional and pulmonary inflammatory changes, were prevented or attenuated by inhibition of microglia activation with not only, intraperitoneal but also, intracerebroventricular minocycline. Inhibition of central microglia activation is a prospective therapy for allergic asthma.

## Data Availability Statement

The raw data supporting the conclusions of this article will be made available by the authors, without undue reservation, to any qualified researcher.

## Ethics Statement

The animal study was reviewed and approved by Ethical Committee of the Fudan University School of Basic Medical Sciences (Nos. 20110307-060 and 20170223-073).

## Author Contributions

JW designed the study and prepared the manuscript. DH performed most of the immunofluorescent, Western-blot, and plethysmographic experiments. HC and MZ helped with the preparation of animal model. All authors helped for interpretation of the data and preparation of the manuscript.

## Conflict of Interest

The authors declare that the research was conducted in the absence of any commercial or financial relationships that could be construed as a potential conflict of interest.

## Abbreviations

ACSF: artificial cerebral spinal fluid
AVPNs: airway vagal preganglionic neurons
BALF: bronchoalveolar lavage fluid
BDNF: brain-derived neurotrophic factor
C_dyn_: dynamic compliance of the lungs
CNS: central nervous system
CSF: cerebral spinal fluid
eNA: the external formation of the nucleus ambiguus
GABA: γ-aminobutyric acid
GAPDH: glyceraldehyde-3-phosphate dehydrogenase
IA-AVPNs: inspiratory-activated airway vagal preganglionic neurons
II-AVPNs: inspiratory-inhibited airway vagal preganglionic neurons
KCC2: K^+^-Cl^–^ co-transporter 2
NA: nucleus ambiguus
NKCC1: Na^+^-K^+^-2Cl^–^ co-transporter 1
NTS: nucleus tractus solitarius
OVA: ovalbumin
PEF: peak expiratory flow
PIF: peak inspiratory flow
R_e_: expiratory resistance of the airway
R_i_: inspiratory resistance of the airway.
